# Postoperative Pulmonary Complications in Patients With Transcatheter Tricuspid Valve Implantation—Implications for Physiotherapists

This article has been retracted.

**DOI:** 10.3389/fcvm.2022.904961

**Published:** 2022-05-19

**Authors:** Peng-Ming Yu, Yu-Qiang Wang, Ze-Ruxing Luo, Raymond C. C. Tsang, Oystein Tronstad, Jun Shi, Ying-Qiang Guo, Alice Y. M. Jones

**Affiliations:** ^1^Rehabilitation Medicine Center, Sichuan University West China Hospital, Chengdu, China; ^2^Key Laboratory of Rehabilitation Medicine in Sichuan Province, Chengdu, China; ^3^Department of Cardiovascular Surgery, Sichuan University West China Hospital, Chengdu, China; ^4^Department of Physiotherapy, MacLehose Medical Rehabilitation Centre, Hong Kong, Hong Kong SAR, China; ^5^Department of Physiotherapy, The Prince Charles Hospital, Queensland, QLD, Australia; ^6^Critical Care Research Group, The Prince Charles Hospital, Queensland, QLD, Australia; ^7^School of Health and Rehabilitation Sciences, The University of Queensland, Queensland, QLD, Australia

**Keywords:** tricuspid regurgitation, transcatheter tricuspid valve replacement, pre-habilitation, inspiratory muscle training, physiotherapy, postoperative pulmonary complications (PPCs)

## Abstract

**Objectives:**

To investigate the incidence of postoperative pulmonary complications (PPCs) and short-term recovery after transcatheter tricuspid valve implantation (TTVI).

**Methods:**

A total of 17 patients diagnosed with severe tricuspid regurgitation who received a LuX-valve TTVI were included in this study. Spirometry lung function, maximal inspiratory pressure (MIP), and 6-min walk test distance (6MWD) were recorded. Prior to surgery, patients were stratified into high or low pulmonary risk groups based on published predefined criteria. A physiotherapist provided all patients with education on thoracic expansion exercises, effective cough and an inspiratory muscle training protocol at 50% of MIP for 3 days preoperatively. All patients received standard post-operative physiotherapy intervention including positioning, thoracic expansion exercises, secretion removal techniques and mobilization. Patients were assessed for PPCs as defined by the Melbourne-Group Score-version 2. Clinical characteristics and hospital stay, cost, functional capacity, and Kansas City Cardiomyopathy Questionnaire (KCCQ) heart failure score were recorded at admission, 1-week, and 30-days post-op.

**Results:**

The mean (*SD*) age of the 17 patients was 68.4 (8.0) years and 15 (88%) were female. Pre-surgical assessment identified 8 patients (47%) at high risk of PPCs. A total of 9 patients (53%) developed PPCs between the 1st and 3rd day post-surgery, and 7 of these 9 patients were amongst the 8 predicted as “high risk” prior to surgery. One patient died before the 30 day follow up. Pre-operative pulmonary risk assessment score, diabetes mellitus, a low baseline MIP and 6MWD were associated with a high incidence of PPCs. Compared to those without PPCs, patients with PPCs had longer ICU and hospital stay, and higher hospitalization cost. At 30 days post-surgery, patients without PPCs maintained higher MIP and 6MWD compared to those with PPCs, but there were no significant between-group differences in other lung function parameters nor KCCQ.

**Conclusion:**

This is the first study to report the incidence of PPCs post TTVI. Despite a 3-day prehabilitation protocol and standard post-operative physiotherapy, PPCs were common among patients after TTVI and significantly impacted on hospital and short-term recovery and outcomes. In the majority of patients, PPCs could be accurately predicted before surgery. A comprehensive prehabilitation program should be considered for patients prior to TTVI.

**Clinical Trial Registration:**

[www.ClinicalTrials.gov], identifier [ChiCTR2000039671].

## Introduction

Severe tricuspid valve regurgitation (TR) accounts for over 30% of degenerative valvular disease in people over 60 years in China (1). The impact of TR on functional status and long-term survival is well known (2). Management of people with TR involves pharmacological treatment of associated heart failure and/or tricuspid valve repair or replacement *via* open-heart surgery. However, conventional open-heart tricuspid interventions are associated with high operative mortality and unsatisfactory outcomes (3) and are often only performed as an additional procedure in concert with aortic or bicuspid valve surgery (4).

In recent years, percutaneous tricuspid valve intervention has been facilitated by improved transthoracic and trans-esophageal imaging and the development of transcatheter tricuspid valve repair devices. Successful transcatheter tricuspid valve intervention or implantation (TTVI) was first reported by Schofer et al. (5). TTVI is now considered a viable, minimally invasive alternative intervention to open-heart surgery, especially in high-risk patients (6). In China, the First-in-Man experience of transcatheter tricuspid valve implantation (TTVI) with the LuX-valve was performed in 12 patients in late 2019 (7). At 30-days post-surgery, there were no deaths or cardiovascular complications in this patient cohort.

The incidence of post-operative pulmonary complications (PPCs) after open-heart surgery has been reported as being between 10 and 25% (8). Reports of perioperative complications associated with TTVI have mainly focused on cardiovascular (9, 10), renal and hepatic systems (11) to date, with no studies reporting on PPCs in this population. While the post-surgical survival rate after LuX-valve implantation has been excellent, the respiratory function and quality of life of patients after surgery has not been described.

The role of physiotherapy following surgery has been well established, and there is strong evidence to support the role of pre-operative physiotherapy reducing PPCs in patients after major abdominal (12) and elective cardiac surgery (13). The West China hospital is a hospital in China dedicated to performing TTVI and has an existing pre- and post- operative physiotherapy service. The aim of this observational study was to report the incidence of PPCs, as defined by the Melbourne Group Scale-version 2 (MGS-ver2) (14), in patients after TTVI with the LuX-valve at the West China Hospital. A secondary aim of this study was to investigate the short-term recovery of lung function and quality of life status after TTVI. Information from this study will guide physiotherapists to further optimize management of patients in this surgical population.

## Materials and Methods

### Study Design

This study is registered with ClinicalTrials.gov (ChiCTR2000039671) and approved by the Biomedical Ethics Committee of West China Hospital of Sichuan University (No. 20201064). The study was conducted in strict accordance with the principles of the Declaration of Helsinki (15) and followed the Strengthening of Reporting Observational Studies in Epidemiology (STROBE) guideline (16) for cohort studies.

### Participants

Patients with severe TR receiving medical treatment at the West China hospital were screened for eligibility for TTVI based on the criteria listed in Box 1.

**BOX 1. Inclusion and exclusion criteria for eligibility of TTVI.**

**Table:** 

**Inclusion criteria** 1. age ≥ 50 years 2. severe or greater TR (based on measured vena contracta width and quantitation of effective regurgitant orifice area (EROA) 3. NYHA classification grade III or IV 4. good left ventricular systolic function with left ventricular ejection fraction ≥ 50 5. ability to understand the purpose of the trial and voluntarily participate and sign the informed consent form, and consented to undergo relevant examinations and clinical management **Exclusion criteria** 1. aortic, mitral or pulmonary valve lesions requiring surgical intervention 2. patients with preoperative circulatory instability, 3. presence of severe hepatic and renal failure; 4. patients with cerebrovascular accident, acute peptic ulcer or upper gastrointestinal bleeding within 3 months and unable to receive anticoagulation or antiplatelet therapy; 5. those who are allergic to aspirin, heparin, clopidogrel, nitinol or contrast media; 6. life expectancy ≤ 1 year. 7. those who have not met the study endpoint time frame for participation in other drug or device clinical trials prior to enrollment

*TTVI = transcatheter tricuspid valve implantation; TR = tricuspid regurgitation; NYHA = New York Heart Association.*

### Echocardiographic Assessment

All patients undertook transthoracic echocardiograms following the American Society of Echocardiography standards for echocardiography core laboratories (17). Tricuspid annulus internal diameter was measured to determine the size of the valve to be implanted. The severity of TR was graded according to vena contracta width and effective regurgitant orifice area (18). These echocardiographic measurements were recorded on admission, at 1-week post-op and 30-days post-op follow up.

### Measurements and Procedures

Reports of transthoracic echocardiograms were discussed with the patients and the TTVI procedure recommended to those who met the eligibility criteria listed in Box 1. Patients who consented to surgery were admitted to the West China hospital 3 days prior to the procedure. Upon admission, demographic data were recorded, and all patients were assessed by a physiotherapist. Pre-surgical Physiotherapy interventions included education on effective coughing, thoracic expansion techniques and importance of mobilization after the procedure. All patients underwent a spirometry lung function test, a 6-min walk test (6MWT) conducted following the American thoracic society guideline (19) and an assessment of maximal inspiratory pressure (MIP) (Digi IMT X1, XEEX Co., Ltd., Xiamen, China). All patients were prescribed an inspiratory muscle training (IMT) program using a digital threshold IMT device (Digi IMT X1, XEEX Co., Ltd., Xiamen, China) with training intensity set at 50% of MIP measured on Day 1. This IMT device records the patient’s training sessions and provides continuous feedback to the physiotherapist and the patient. Patients were asked to complete five sets of 10 repetitions per day, with a 1-min interval between each set (20). All training sessions were supervised by the treating physiotherapist. The intensity of the IMT exercise was monitored *via* a Rate of Perceived Exertion (RPE) scale, with patients asked to exercise at moderate intensity (5–6/10). The patients also completed the Kansas City Cardiomyopathy Questionnaire (KCCQ). All pre-operative assessment procedures were repeated 1-week post-surgery and during their 30-day follow up. All patients were assigned a “high” or “low” pre-operative pulmonary risk score according to a previously validated pre-operative pulmonary risk assessment tool (Box 2) (21).

**BOX 2. Pre-operative pulmonary risk assessment.**

**Table:** 

Items	Points
Age > 70 years	1
Cough and expectoration	1
Diabetes mellitus	1
Smoker	1
Chronic obstructive pulmonary disease	1
FEV_1_ < 75% predicted or pulmonary medication used	1
Body mass index > 27	1
FEV_1_ < 80% predicted and FEV_1_/FVC < 70% predicted	2
Total points	
Low risk = 0 or 1 point; High risk = 2 or more points	

### Transcatheter Tricuspid Valve Implantation

The procedure was performed under general anesthesia. A small (5–8 cm) intercostal incision was made at the fourth intercostal space on the right side of the chest. The location of the right atrium was identified by transesophageal echocardiography and fluoroscopy (Figure 1A). After the right atrium was revealed, a catheter sheath was then placed through the right atrium; and right atrial pressure, right ventricular pressure and pulmonary artery pressure measured *via* a cardiac catheter. Assisted by contrast filling the right ventricular cavity, the tricuspid annulus position was determined. The LuX- valve (Figure 2), a prosthetic valve made from bovine pericardium, composed of an umbrella disc stent, an interventricular septal anchor, and two expanded polytetrafluroethylene-covered graspers, was “delivered” through the tricuspid orifice and anchored to the annulus and atrial wall tissue (7). The valve position, any perivalvular leakage and orifice regurgitation were checked by TTE (Figures 1B–I). All patients were managed post-operatively in the intensive care unit (ICU) until stability of cardiovascular and pulmonary function was achieved. The grading of tricuspid regurgitation and paravalvular leak of the implanted valve was monitored by Doppler cardiac ultrasound (Figure 3).

**FIGURE 1:** TTVI procedure: After a small (5–8 cm) intercostal incision was made in the fourth intercostal space on the right side of the chest, the location of the right atrium was identified by transesophageal echocardiography and fluoroscopy **(A)**. Digital subtraction angiography (DSA) was used to reveal the contrast medium flow between the right atrium and ventricle. **(B)** Shows the back flow of contrast medium from the right ventricle into the right atrium before LuX-valve implantation. Under DSA and transthoracic echocardiogram guidance, the valve was loaded into the delivery system and passed through the tricuspid orifice toward the right ventricular cavity **(C)**. Interventricular anchorage, parallel to the septum was assured **(D)**. The anterior valve hook-and-jaw device was gradually released and hooked onto the anterior valve leaflet, after the valve position was determined **(E)**. The atrial facet umbrella disc was released **(F)**. Transthoracic echocardiogram confirmed the position of umbrella disc in the annulus and atrial wall tissue, and ensured there was no obvious paravalvular leakage **(G)**. The valve was finally released when the septal anchoring device was in position **(H)**. After LuX-valve implantation, DSA showed satisfactory right ventricular filling with no or minimal, contrast medium back-flow **(I)**.

**FIGURE 2:** The LuX-valve. The LuX-valve has 4 components: (1) a bovine-pericardium prosthetic tricuspid-valve pre-treated with the JeniGal anti-calcification process; (2) an umbrella disc stent made up of a self-expanding nickel-titanium alloy, for attachment to the atrial surface or tricuspid-annulus. The nickel-titanium frame is laser-cut, heat and surface treated so that it can be easily compressed, while providing adequate strength, durability and flexibility during deployment. Once the frame is deployed at the target location in the heart, it self-expands into its memorized, predesignated shape after warming to body temperature; (3) an interventricular anchorage to the septum; and (4) 2 expanded polytetrafluoroethylene-covered anchoring pins to fix the leaflets and further stabilize valve anchorage. Photo reproduction authorized by Jenscare Scientific Co., Ltd.

**FIGURE 3:** Pre and post-surgery Doppler echocardiograpy. **(A)** Preoperative cardiac ultrasound showing a large back flow from the right ventricle to the right atrium; **(B)** postoperative cardiac ultrasound showing no back-flow from the right ventricle to the right atrium.

### Post-operative Procedures

All patients received physiotherapy management as indicated. Physiotherapy interventions were delivered according to assessment findings and included positioning, thoracic expansion exercises, secretion removal techniques and mobilization. All patients were observed for signs of PPCs from Day 1 post-surgery, following the MGS-ver2 (14). When 4 of the 8 diagnostic criteria were present, a diagnosis of PPC was confirmed. The cost of hospital stay for all patients was recorded from the patients’ hospital invoice.

### Statistical Analyses

All data analyses were conducted using IBM SPSS for Windows, version 25.0 (Armonk, NY: IBM Corp.). The data were checked for completeness and normality with the Shapiro-Wilk test. In the case of a missing value, for example if a patient failed to participate in the reassessment, the case was excluded from analysis. Descriptive statistics of nominal or dichotomous variables were shown as counts and percentages. As the sample size was small, data for continuous variables were displayed as median, 25th and 75th percentiles. The primary outcome of interest was the development of PPCs as defined by the MGS-ver2. Characteristics of patients were compared between those with PPCs (PPC group) and without PPCs (non-PPC group) using the Fisher’s exact test for nominal variables and Mann-Whitney U test for continuous variables. The secondary outcomes, New York Heart Association (NYHA) classification, TR severity, lung function, 6-min walk distance (6MWD), and KCCQ score at different time points were analyzed using the Friedman test to illustrate the trend of changes in both groups. Duration of hospitalization and cost were compared between the two groups with the Mann–Whitney *U*-test. All statistical tests were two-tailed with the level of significance set at 0.05.

## Results

A total of 19 patients were evaluated from October 2020 to March 2021 and considered eligible for the LuX-Valve procedure. Seventeen of these 19 patients consented to have surgery, with all 17 consenting to participate in this study. Eight patients were stratified as having a high risk of pulmonary complications based on their pre-operative pulmonary risk score (21). Demographic data and clinical characteristics of the consenting patients are listed in Table 1. Factors which contributed to the pulmonary risk score for each patient are displayed in Table 2.

**TABLE 1:** Demographic and patient clinical characteristics recorded on admission.

Patient characteristics (*n* = 17)	Median or *n*	(Q1–Q3) or (%)
Age, y	68	(62–74)
Female	15	(88)
BMI	23.8	(20.9–26.7)
Smoking history	2	(12)
Smoker Non-smoker Ex-smoker	2 15 0	(11.8) (88.2) (0)
History of median sternotomy	12	(71)
**Comorbidity**		
COPD	8	(47)
Atrial fibrillation	14	(82)
Type 2 diabetes	5	(29)
Hypertension	4	(24)
Coronary arterial disease	1	(6)
Left ventricular ejection fraction (%)	61	(58.5–64.5)
Pulmonary arterial pressure, mmHg	36	(32.0–44.5)
EuroSCORE	7	(6–9)
Pulmonary risk		
High	8	(47)
Low	9	(53)
**NYHA classification**		
III	16	(94)
IV	1	(6)
**TR severity**		
Severe	9	(53)
Massive	6	(35)
Torrential	2	(12)

*PPCs, postoperative pulmonary complications; BMI, body mass index; COPD, chronic obstructive pulmonary disease; EuroSCORE, European system for cardiac operative risk evaluation; NYHA, New York Heart Association; TR, tricuspid regurgitation.*

*Data in median (Q1–Q3) or n (%).*

**TABLE 2:** Scoring of pre-operative pulmonary risk assessment in the 17 patients consented for surgery.

Patient	Contributing factors of pulmonary risk scoring								Total risk score	Pulmonary risk	* PPCs
	
	Age > 70	C&E	DM	Sm	COPD	FEV_1_ & med	BMI > 27	FEV_1_/FVC			
1	1	1	0	1	1	0	0	0	4	High	Yes
2	0	0	0	0	0	0	0	0	0	Low	Yes
3	0	0	0	0	1	0	0	0	1	Low	Yes
4	1	1	0	0	1	0	0	0	3	High	Yes
5	0	0	0	0	1	0	0	0	1	Low	−
6	1	0	1	0	0	0	0	0	2	High	Yes
7	0	0	1	0	0	1	0	1	4	High	Yes
8	0	0	0	0	0	0	1	0	1	Low	−
9	0	0	0	0	1	0	0	0	1	Low	−
10	1	0	0	0	0	1	0	1	4	High	−
11	1	0	0	0	0	0	0	0	1	Low	−
12	0	0	0	0	1	0	0	0	1	Low	−
13	0	0	0	0	0	0	1	0	1	Low	−
14	0	1	1	1	1	1	0	0	5	High	Yes
15	0	0	1	0	1	0	1	0	3	High	Yes
16	0	1	1	0	0	1	1	1	6	High	Yes
17	1	0	0	0	0	0	0	0	1	Low	−

0, No; 1, Yes; C&E, cough and expectoration; DM, diabetes mellitus; Sm, smoker; FEV1 & med, FEV_1_ < 75% predicted/pulmonary medication use; FEV1/FVC, FEV_1_ < 80% predicted and FEV_1_/FVC < 70% predicted; PPC, post-op pulmonary complication; *Yes, those who developed PPC.

Three patients had a permanent pacemaker for 1–3 years prior to the TTVI procedure. None of these patients required pacemaker post-surgery and all patients remained pacemaker free 30 days post-surgery. One patient suffered an exacerbation of severe heart failure after discharge to home and died on post-operative day 17. At 1-week post-surgery, one patient (patient 6) was found to have severe paravalvular leak as well as symptoms of hypoperfusion. Tricuspid valvuloplasty under open-sternotomy was performed. The prosthetic valve was found to be structurally normal, but the septal anchoring device had detached from the septum and a cleft was observed between the prosthetic valve holder and the tricuspid septal annulus. Surgical sutures were used to reinforce the valve loosening site. Postoperative echocardiography suggested the perivalvular leak had decreased. At the 30-days postoperative follow-up, the patients’ heart failure symptoms had improved but she continued to need respiratory support in ICU.

At the 30-day follow up, one patient remained bed-bound (due to gastrointestinal bleeding), one failed to attend the assessment and one patient had thrombosis detected at the tricuspid valve by ultrasound and was instructed by the medical practitioner to stay at home. Consequently, only 13 patients completed the 30-days follow-up assessments.

### Post-operative Complications

A total of 9 patients (53%) developed PPCs based on MGS-ver2. Table 3 displays the factors that contributed to the diagnosis of PPCs in each patient. Seven of these 9 patients were correctly predicted to have a PPC. Only one patient that was predicted to have a high risk of PPCs prior to the surgery did not end up having a PPC. PPCs were observed on day 1 post surgery for 5 patients, day 2 for 2 patients and day 3 for 2 patients (Table 3). Five of these 9 patients (56% of those with PPCs) were diagnosed with pneumonia, 3 with atelectasis (33%) and 1 with pleural effusion (11%). Of the 5 patients diagnosed with pneumonia, 1 also had a pneumothorax and another had a pleural effusion as well. A total of 5 patients required mechanical ventilation for more than 48 h. Of the patients diagnosed with pneumonia, bacterial cultures (klebsiella, enterobacter cloacae, aspergillus flavus) were observed in 3, but no bacteria were cultured in the other 2 patients. Nearly all patients (16. 94% of the total cohort) exhibited an elevated white cell count with 13 (76%) having abnormal breath sounds on auscultation which differed from their pre-operative assessment and 11 (65%) showing chest radiographic changes.

**TABLE 3:** Identification of pulmonary complications using the MGS-ver 2 in patients after TTVI.

Patient number	Factors in Melbourne group scale (MGS)-version 2								PPC identified	Post-op date identified	Medical pulmonary diagnosis	Pre-op pulmonary risk
	
	1	2	3	4	5	6	7	8				
1*	x			x	x			x	Yes	3	Pleural effusion, MV > 48 h	High
2	x	x		x	x	x	x	x	Yes	1	Pneumonia (Klebsiella), MV > 48 h	Low
3	x	x			x	x	x	x	Yes	2	Pneumonia (no bacteria cultured)	Low
4	x			x	x	x	x	x	Yes	1	Pneumonia (no bacteria cultured), MV > 4 h	High
5	x				x				No		−	Low
6	x			x	x	x	x	x	Yes	3	Pneumonia (Aspergillus flavus), Pneumothorax MV > 48 h (in ICU at day 7, in bed at 30 days)	High
7	x	x	x	x	x	x	x	x	Yes	2	Pneumonia (Enterobacter cloacae), Pleural effusion MV > 48 h (in ICU at day 7, did not FU at 30 days)	High
8					x				No		−	Low
9					x				No		−	Low
10	x				x			x	No		−	High
11					x			x	No		−	Low
12				x	x				No		−	Low
13								x	No		−	Low
14	x	x			x			x	Yes	1	Atelectasis	High
15	x	x	x		x			x	Yes	1	Atelectasis (thrombosis at follow up)	High
16	x	x		x	x			x	Yes	1	Atelectasis	High
17					x			x				Low
Total	**11**	**6**	**2**	**7**	**16**	**5**	**5**	**13**				

*TTVI, transcatheter tricuspid implantation; PPC, Post-operative pulmonary complication; MGS-ver2, Melbourne Group Scale ver2; MV, mechanical ventilation.*

Factor #: 1, chest radiograph report of consolidation/collapse; 2, raised temperature > 38^°^C on two or more consecutive days; 3, SpO_2_ < 90% on room air on two consecutive days (SpO_2_, pulse oximetry saturation of oxygen); 4, production of yellow or green sputum which is different to pre-operative assessment; 5, an otherwise unexplained white cell count > 11 × 10^9^L^–1^ or prescription of an antibiotic specific for respiratory infection; 6, physician diagnosis of chest infection; 7, presence of infection on sputum culture report; 8, abnormal breath sounds on auscultation which differ from pre-operative assessment *died at post-op day 17.

### Characteristics of Patients With and Without Post-operative Complications

Table 4 displays all measured outcomes recorded in patients with and without PPCs. The main differences in characteristics between the patients who had PPCs vs. those who did not were a higher incidence of type 2 diabetes mellitus as comorbidity (55.6% vs. 0%, *p* = 0.03) and high pre-operative pulmonary risk score (77.8% vs. 12.5%, *p* = 0.02), and a lower % predicted MIP (62.02 cmH_2_O vs. 95.87, *p* = 0.04) and shorter 6MWD (215.5 vs. 345 m, *p* = 0.01). Patients with PPCs had a significantly longer length of ICU stay (median 72 vs. 20.5 h, *p* < 0.01), longer length of hospital stay (median 11 vs. 7.5 days, *p* < 0.01), and higher hospital costing (median 74,300 vs. 52,000 Yuan, *p* < 0.01) (Table 4).

**TABLE 4:** Outcome comparisons for patients with and without post-operative complications.

	PPC group (*n* = 9)	Non-PPC group (*n* = 8)	*P*-value
	
	Median (Q1–Q3) or *n* (%)		
Age, years	67.0 (61.5–78.0)	70.0 (63.0–73.5)	0.74
Female, *n*(%)	7 (77.8)	8 (100)	0.47
BMI, kg/m^2^	22.1 (20.4–26.7)	25.1 (23.4–27.3)	0.39
Smoker, *n*(%)	2 (22.2)	0 (0)	0.47
Median sternotomy, *n*(%)	7 (77.8)	5 (62.5)	0.62
**Comorbidity,** *n*(%)			
COPD	5 (55.6)	3 (37.5)	0.64
Atrial fibrillation	7 (77.8)	7 (87.5)	>0.99
Type 2 diabetes	5 (55.6)	0 (0)	0.03
Hypertension	1 (11.1)	3 (37.5)	0.29
Coronary arterial disease	0 (0)	1 (12.5)	0.47
Renal insufficiency	3 (33.3)	1 (12.5)	0.58
Peripheral arteriosclerosis	3 (33.3)	4 (50.0)	0.64
Stroke	1 (11.1)	0 (0)	>0.99
Hyperlipidemia	2 (22.2)	1 (12.5)	>0.99
Inspiratory muscle weakness	4 (44.4)	0 (0)	0.08
Pulmonary arterial hypertension	7 (77.8)	4 (50.0)	0.34
Peripheral edema	6 (66.7)	6 (75.0)	> 0.99
Left ventricular ejection fraction,%	62.0 (58.5–64.5)	60.5 (58.5–64.8)	0.81
Pulmonary arterial pressure, cmH_2_O	32.0 (30.5–48.5)	36.0 (35.0–40.0)	0.59
EuroSCORE	7.0 (6.5–9.5)	8.5 (6.0–9.0)	0.92
Pulmonary risk, *n* (%)			
High	7 (77.8)	1 (12.5)	0.02
Low	2 (22.2)	7 (87.5)	
**NYHA classification on admission 7, *n* (%)**			
III	8 (88.9)	8 (100)	>0.99
IV	1(11.1)	0(0)	
**NYHA classification at 1-week post-op, *n* (%)**			
I	4 (44.4)	8 (100)	0.10
II	1 (11.1)	0 (0)	
III	3 (33.3)	0 (0)	
IV	1 (11.1)	0 (0)	
NYHA classification at 30-days post op, *n* (%)*			
I	2 (28.6)	2 (25.0)	0.33
II	3 (42.9)	5 (62.5)	
III	0 (0)	1 (12.5)	
IV	2 (28.6)	0 (0)	
**TR severity on admission, *n* (%)**			
None	0 (0)	0 (0)	0.70
Mild	0 (0)	0 (0)	
Moderate	0 (0)	0 (0)	
Severe	4 (44.4)	5 (62.5)	
Massive	4 (44.4)	2 (25.0)	
Torrential	1 (11.1)	1 (12.5)	
**TR severity at 1-week postop, *n* (%)**			
None	3 (42.9)	1 (12.5)	0.50
Mild	4 (44.4)	6 (75.0)	
Moderate	1 (11.1)	1 (12.5)	
Severe	1 (11.1)	0 (0)	
Massive	0 (0)	0 (0)	
Torrential	0 (0)	0 (0)	
TR severity at 30-days post-op, *n* (%)*			
None	2 (28.6)	1 (12.5)	0.55
Mild	3 (42.9)	5 (62.5)	
Moderate	1 (14.3)	2 (25.0)	
Severe	1 (14.3)	0 (0)	
Massive	0 (0)	0 (0)	
Torrential	0 (0)	0 (0)	
**Lung function on admission**			
% Predicted FEV_1_	92.8 (80.5–120.9)	86.0 (81.7–94.0)	0.75
% Predicted FVC	106.2 (82.6–123.7)	91.0 (86.7–96.1)	0.75
MVV, l/min	55.8 (47.8–67.2)	55.6 (48.9–59.2)	0.60
% Predicted MIP, cmH_2_O	62.02 (55.22–83.89)	95.87 (87.29–108.73)	0.04
**Lung function at 1-week post-op**			
% Predicted FEV_1_	105.6 (88.1–144.4)	91.2 (85.4–107.1)	0.57
% Predicted FVC	117.3 (88.0–134.0)	99.0 (92.0–108.2)	0.75
MVV, l/min	57.8 (52.1–69.1)	65.4 (53.2–66.7)	0.34
% Predicted MIP, cmH_2_O	64.32 (60.35–85.56)	102.53 (91.88–114.85)	0.03
Lung function at 30-days post-op *			
% Predicted FEV_1_	97.5 (80.3–113.8)	92.0 (88.0–97.0)	0.32
% Predicted FVC	95.3 (83.7–114.1)	90.9 (78.6–101.6)	0.39
MVV, l/min	50.3 (38.3–68.2)	56.7 (51.3–63.4)	0.48
% Predicted MIP, cmH_2_O	58.29 (54.99–94.54)	104.13 (97.20–120.98)	0.03
**6-min walk distance, m**			
On admission	215.5 (125.0–349.5)	345.0 (327.8–384.8)	0.01
At 1-week post-op^#^	234.5 (177.0–336.3)	315.5 (259.5–405.8)	0.17
At 30 days post-op^##^	273.0 (232.5–353.3)	353.0 (307.8–464.5)	0.04
**KCCQ score**			
On admission	42.5 (27.1–71.6)	61.1 (42.5–75.4)	0.07
At 30-days post-op*	60.0 (42.9–78.3)	64.2 (45.0–69.2)	0.20
Duration of surgery, min	123.0 (105.0–130.0)	100.0 (92.0–138.8)	0.44
Duration of MV, hours	52.0 (14.5–63.5)	16.0 (13.2–18.8)	0.09
Length of ICU stay, hours	72.0 (45.5–95.0)	20.5 (16.0–22.8)	<0.01
Length of POS, days	11.0 (10.0–17.0)	7.5 (7.0–8.0)	0.01
Hospital Costing, thousands yuan	74.3 (65.2–210.2)	52.0 (49.5–57.5)	<0.01

*PPCs, postoperative pulmonary complications; BMI, body mass index; COPD, chronic obstructive pulmonary disease; NYHA, New York Heart Association; TR, tricuspid regurgitation, KCCQ, Kansas City Cardiomyopathy Questionnaire; MV, mechanical ventilation; POS, post-op hospital stay.*

*Two patients from the PPC group failed to attend the assessment (1 patient died and 1 failed to attend assessment).

*^#^Five patients from the PPC group failed to participate at week 1 post-surgery (2 in ICU, 3 on wheelchair).*

*^##^Four patients from the PPC group failed to participate in 6MWT at 30-days post-surgery (1 died, 1 failed to attend, 1was diagnosed with thrombosis requested by doctor to stay at home and 1 still restricted to bed mobility).*

### Secondary Outcomes—Tricuspid Valve Regurgitation Severity, New York Heart Association Classification, Lung Function, 6-Min Walk Test Distance and Kansas City Cardiomyopathy Questionnaire

At 1-week post-surgery, five patients were unable to participate in the 6MWT (reasons listed in Table 4); by 30-days after surgery, four patients were still unable to complete a 6MWT. Two of these patients also failed to attend the assessment of TR, NYHA, KCCQ, and lung function assessment. These patients were all in the PPC group. Consequently, there were only 7 patients available for trend analysis in the PPC group, and information on post-operative 6MWD was only available from four patients in this group. Prior to surgery, two patients had torrential TR and the other 15 had either severe or massive TR. Significant reduction in TR severity was observed in both groups (Table 5), but no between group differences were observed.

**TABLE 5:** Trend analysis of NYHA classification, TR severity, lung function, 6MWD, and KCCQ. Analysis by Friedman test.

Variables	PPC group		No-PPC group	
		
	*P*-value	*n*	*P*-value	*n*
NYHA classification	0.26	7	<0.01	8
TR severity	<0.01	7	<0.01	8
% predicted FEV_1_	<0.01	7	0.02	8
% predicted FVC	0.02	7	<0.01	8
MVV	0.12	7	<0.01	8
% predicted MIP	0.51	7	0.03	8
6MWD	0.09	4	0.21	8
KCCQ	1.00	7	1.00	8

*NYHA, New York Heart Association; TR, tricuspid regurgitation; FEV1, forced expiratory volume in 1 s; FVC, forced vital capacity; MVV, maximal voluntary ventilation; MIP, maximal inspiratory pressure; 6MWD, 6 min walk distance; KCCQ, Kansas City cardiomyopathy questionnaire; n, number of patients completed full trend analysis.*

Reduction in number patients with NYHA classification of III and IV was observed in both groups over time (from 9 to 2 in the PPC group and 8–1 in the non-PPC group), but there was no between-group difference at the various time points (Table 4). Trend analysis revealed that improvement over time reached a statistically significant level in the non-PPC group only (*p* < 0.01, Table 5).

Lung function changes were similar for both groups except the % predicted MIP being higher in the non-PPC group at all-time points (*p* < 0.05, Table 4). Significant improvement in all lung function parameters over time was observed in the non-PPC group, but improvement of % predicted FEV_1_ and % predicted FVC was also observed in the PPC group (Table 5).

Patients in the non-PPC group exhibited a higher 6MWD at baseline compared to the PPC group (345 vs. 215.5 m) and also at 30-days post-surgery (353 vs. 273 m) (Table 4). Both groups demonstrated some improvement over time, but the changes did not reach a statistically significant level (Table 5).

There were no between-group differences in KCCQ score at baseline or at 30-days post-surgery. The change over time was not significant in either group (Table 5).

## Discussion

To the authors knowledge, this is the first study that reports the incidence of PPCs after TTVI. This study shows that PPCs, as defined by the MGS-ver2, occurred in 53% of patients following TTVI and manifested within the first 3 days post-surgery. Not surprisingly, patients who experienced PPCs required significantly longer duration of mechanical ventilation, had longer duration of stay in ICU and in hospital, and consequently had a higher cost of their hospital admission (Table 4). It has previously been reported that the cumulative reported incidence of PPCs in cardiac surgery with cardiopulmonary bypass varied from 10 to 25% (8). Comparisons between the results of the current study and studies reporting on patients undergoing cardiac surgery requiring median sternotomy and cardiopulmonary bypass is not relevant as the patients in this study did not require cardiopulmonary bypass and median sternotomy, which are associated with post-operative lung injuries and PPCs (22). However, despite not undergoing median sternotomy and cardiopulmonary bypass, the incidence of PPCs in our cohort was higher than previously reported. We postulate that this is because our study cohort all had severe, massive, and even torrential TR, and the majority (78% in the PPC group and 50% in the non-PPC group) had pulmonary hypertension (Table 4). Severe TR has been shown to be associated with decreased survival (2) and patients with pulmonary hypertension, particularly in association with right ventricular dysfunction, have been shown to be more prone to hypoxemia and circulatory failure following complex surgery (23). More patients in the PPC group had worse TR associated with pulmonary hypertension, than in the non-PPC group. This may explain the high incidence of PPCs in our TTVI cohort in comparison with those reported after conventional cardiac surgery (8).

### Risk Factors and Prediction of Post-operative Complications

Analysis of patient characteristics between those with or without PPCs showed that the patients who were more likely to develop PPCs were those with diabetes mellitus (DM), high pre-operative pulmonary risk assessment scores, a lower MIP [expressed as % predicted of matched gender and age (24)] and lower 6MWD prior to surgery (Table 3). DM has previously been demonstrated as a risk factor for developing PPCs after cardiac surgery (25). Patients with DM after off-pump coronary artery bypass graft were found to have longer ICU stays and greater incidence of infection than those without DM (25).

In our patient cohort, 8 patients were found to have a high pulmonary risk-score before their procedure with 7 of them developed PPCs, and all patients with DM had PPCs. This suggests that specific attention, such as close perioperative blood-glucose control (25), should be considered an essential part of a prehabilitation/pre-surgical optimization program. Further, as 7 of the 9 patients who developed PPCs were correctly predicted by the pre-operative pulmonary risk assessment tool (21), this suggests that there is a good opportunity for those likely to experience PPCs to be identified well before TTVI, and subsequently a specific prehabilitation and rehabilitation pathway could be proactively planned for this population. This may include intensive pre-operative IMT, extra education regarding thoracic expansion exercise commencing immediately upon regaining consciousness after surgery (26), extubation directly to high flow oxygen therapy or non-invasive ventilation (NIV), early physiotherapy review and potentially a greater focus on positioning/mobility/breathing exercises with an aim to optimize lung expansion and focus on prevention of atelectasis. Nursing staff should be educated and empowered to ensure these strategies (especially deep breathing exercises) are commenced as soon as possible.

Poor % predicted MIP on admission was also one of the possible predictors for PPCs (Table 4). The role of pre-operative physiotherapy in reduction of PPCs has been well established in patients after major abdominal (12) as well as elective cardiac surgery (13), with multiple studies demonstrating the effectiveness of pre-operative IMT in improving MIP and reducing post-operative PPCs (27). All patients in our cohort were admitted to the hospital 3 days prior to their procedure, and during the period before their procedure they received pre-operative physiotherapy intervention consisting of education on lung expansion exercises and effective coughing technique, and they were given a 3-day protocol of IMT. However, previous studies have suggested that meaningful improvements in MIP resulted after a training duration of 5–14 days (27, 28), so it is likely that the time available for this intervention was not sufficient to prevent PPCs.

Apart from meeting the MGS-ver2 criteria for PPCs, these patients were also diagnosed medically with “recognized” pulmonary complications, including pneumonia, pleural effusion, pneumothorax, atelectasis, and respiratory failure that required mechanical ventilation for over 48 h (29). Evaluation of the patients’ scoring profile of MGS-ver2 showed that 6 of the 7 patients who had productive cough prior to surgery developed PPCs (Table 3), and 5 of these 6 patients were diagnosed with pneumonia. Pleural effusion and pneumothorax cannot be prevented by pre-operative physiotherapy, but it appears that a 3-day prehabilitation period perhaps was too short to sufficiently prepare these patients to fully ameliorate the risk of post-operative pneumonia. Chest infection acquired before surgery was associated with worse (reported odds ratio of 5.5) post-operative pulmonary outcomes, including respiratory failure, pulmonary atelectasis, and pleural effusion (30). China has a high incidence of community acquired pneumonia (CAP) (31), but unfortunately no data were collected in this study to explain any possible relationship between PPCs and CAP.

### Trend of Physical Function Recovery After Transcatheter Tricuspid Valve Implantation

A majority of the TTVI patients were significantly deconditioned (NYHA class III or IV) and all endured either a severe, massive or torrential degree of tricuspid regurgitation (Table 1). The 6MWD recorded prior to surgery by patients who developed PPCs was 215 m, which was significantly lower than that covered by patients who did not develop PPCs (345 m) (Table 4). This finding corresponds with other studies having demonstrated that a 6MWD < 300 m is associated with poorer outcomes (32, 33). Further, a poor pre-operative 6MWD has been shown to be associated with a higher incidence of PPCs (34), therefore cardiovascular endurance and strengthening exercises should be considered for inclusion in the prehabilitation program to maximize patients’ functional capacity prior to surgery. However, the safe intensity levels and optimal duration required to achieve a meaningful improvement in physical capacity pre-operatively in this high-risk population of severe TR remains to be determined. While this study showed a significant trend in improvement in TR severity for all patients, improvement in NYHA classification and lung function over time was demonstrated only in patients without PPCs. In accord with other studies on patients post TTVI (35, 36), our patients demonstrated similar improvement in 6MWD and KCCQ score over time, however, the improvement did not reach a statistically significant level in our cohort. Nevertheless, our data must be interpreted cautiously, as only 13 patients completed the 30-days reassessment and five patients were unable to conduct the 6MWT at week 1, these missing data further reduce the power of the already small sample size. All missed assessments were from patients in the PPC group, thus the recovery pattern of patients with PPCs warrant further investigation.

### Duration of Intensive Care Unit Stay

In accord with other reports (37), PPCs led to increased duration of stay in ICU and hospital and economic burden. In our patient cohort, the median hospital cost for those with PPCs was ¥74,300 Chinese Yuan, equivalent to US $12,000. The median hospital cost for those without PPCs was only ¥52,000 (US$8,000); this difference in cost is very significant for the patients, with hospital fees in China commonly paid for by the patients; it should be noted that the reported average annual income in China in 2021 was ¥35,128 (US$5,404) (38). Therefore, any strategies that can reduce the incidence of PPCs will not only deliver better patient outcomes and reduce hospital and ICU length of stay, but will also have significant financial benefits for the patients and their families.

### Future Studies

The physiotherapist is an essential member of the health care team and plays an important role in prevention of post-operative complications and to maximize recovery, but there is currently no recommended “gold-standard” physiotherapy care before or after TTVI. The findings of this study suggests that patients, particularly those with DM, productive cough and MIP and 6MWD below normal values of matched gender and age, should receive an individualized and targeted prehabilitation program which includes comprehensive education, intensive IMT training, and cardiovascular endurance and strengthening exercises that improves physical capacity prior to their procedure. Such a program could be home or hospital based, prescribed by a physiotherapist, and commenced as early as possible prior to surgery to allow sufficient time for an optimal outcome. It should be noted that the concepts of pre-operative physiotherapy training and education are only just developing in various provinces in China. Therefore further investigation is required to determine not only the optimal training duration and intensity, but what the program should consist of as well as what mode of delivery is required for an effective pre-operative physiotherapy program in this patient cohort. This study suggests IMT training of 3 days duration prior to surgery and using the protocol utilized in this study may not be sufficient to prevent PPCs. Previous studies have suggested that pre-operative IMT of at least 5 days duration is necessary to achieve an effective reduction in the PPC rates (28). More studies are warranted on feasibility and safety, as well as comparing the outcomes of various modes of physiotherapy intervention, such as general rehabilitation with varying intensity of IMT.

### Limitations of the Study

There are several limitations of this study that affect interpretation of the findings. This study was not intended to be an interventional study. The study aimed to observe the incidence of PPCs in patients after TTVI. A true observational study should not be “contaminated” by the addition of an intervention, however these patients received pre-operative physiotherapy care. It could be validly argued that any physiotherapy intervention might have influenced the rate of PPCs. However, the physiotherapy intervention adopted in this study was standardized for all patients and our protocol reflected recommended TTVI management. Although a trend of improvement from pre-operative baseline measures of MIP, 6MWD and KCCQ score was apparent in our patient cohort in the 1-week and 30-day post-operative follow up, we are unable to determine whether the rate of PPCs or post-operative pulmonary and functional improvement was influenced by the presence and/or intensity of physiotherapy intervention. However, one important finding which emerged from this study was that the cohort of patients who did not develop PPCs had a higher pre-operative MIP and 6MWD and did not have a productive cough.

Another limitation of this study is the small sample size, however, TTVI is a novel intervention in China and patient acceptance is limited. The third limitation of this study was that we were only able to speculate on the reasons for the high rate of pneumonia in our patient cohort. The incidence of CAP in China is high and varies across different regions. We did not investigate the past incidence of pneumonia and acknowledge that this could have made TTVI patients more susceptible to post-operative pulmonary infection.

## Conclusion

This study showed that despite a 3-day prehabilitation protocol and standard post-operative physiotherapy, PPCs were common among patients after TTVI. PPCs can be accurately predicted pre-surgery, and a comprehensive prehabilitation program should be considered for patients identified with a high pre-operative pulmonary risk score, diabetes mellitus, low MIP and 6MWD prior to TTVI. Similarly, these patients should receive more intensive interventions aimed at reducing the risk and impact of PPCs after their procedure.

## Data Availability Statement

The raw data supporting the conclusions of this article will be made available by the authors, without undue reservation.

## Ethics Statement

The studies involving human participants were reviewed and approved by the Biomedical Ethics Committee of West China Hospital of Sichuan University (No.20201064). The patients/participants provided their written informed consent to participate in this study.

## Author Contributions

P-MY and Y-QW conceived, designed, planned the study, and interpreted results. P-MY contributed to acquisition, analysis, and interpretation of data. P-MY, Y-QG, and AJ drafted the report. P-MY, Y-QW, Z-RL, RT, OT, and AJ involved in the critical revision of the manuscript. RT and JS contributed to statistical analysis. Y-QG and P-MY contributed to administrative, technical, and material support. All authors contributed to the article, data acquisition, and approved the submitted version.

## Conflict of Interest

The authors declare that the research was conducted in the absence of any commercial or financial relationships that could be construed as a potential conflict of interest.

## Publisher’s Note

All claims expressed in this article are solely those of the authors and do not necessarily represent those of their affiliated organizations, or those of the publisher, the editors and the reviewers. Any product that may be evaluated in this article, or claim that may be made by its manufacturer, is not guaranteed or endorsed by the publisher.
